The article "Wilson Disease Masquerading as Nephrotic Syndrome: A Case Report" was published in 2025. Journal: Cureus.

# Wilson Disease Masquerading as Nephrotic Syndrome: A Case Report

**DOI:** 10.7759/cureus.86250

**Published:** 2025-06-17

**Authors:** Gaurav Gupta, Shabnam Kalita, Himel Mondal, Jaya Shankar Kaushik

**Affiliations:** 1 Pediatrics, All India Institute of Medical Sciences, Guwahati, IND; 2 Physiology, All India Institute of Medical Sciences, Deoghar, IND

**Keywords:** ascites, kayser-fleischer ring, kf ring, nephrotic-range proteinuria, nephrotic syndrome, portal hypertension, wilson disease

## Abstract

Wilson disease (WD) is a rare, autosomal recessive disorder characterized by defective copper metabolism. Renal manifestations in WD are uncommon, and nephrotic syndrome as an initial presentation is rare. An eight-year-old boy presented with progressive abdominal distension and decreased urine output. Examination revealed pedal edema, ascites, and icterus. Investigations showed nephrotic range proteinuria, elevated liver enzymes, low serum ceruloplasmin, and Kayser-Fleischer rings, confirming a diagnosis of WD with associated nephrotic syndrome. WD presented with nephrotic syndrome and was confirmed by clinical findings, biochemical tests, and slit-lamp examination. The patient was started on oral penicillamine, zinc supplementation, hepatic support, and a copper-restricted diet. Subsequent follow-up showed symptomatic and biochemical improvement. Resolution of ascites and proteinuria was achieved, with stabilization of liver function. The patient was later managed for portal hypertension with spironolactone and propranolol. Hence, nephrotic syndrome can be a rare presenting feature of WD. Early recognition and multidisciplinary management are essential for favorable outcomes.

## Introduction

Wilson disease (WD) is an inherited, autosomal recessive disorder due to an ATP7 B gene mutation, resulting in defective copper metabolism and leading to progressive hepatolenticular damage [1]. ATP7 B is involved in copper transportation within the cells and its excretion after being incorporated into ceruloplasmin through bile. A mutation in this gene leads to excess free copper in the liver, brain, and other organs, which may either cause direct toxic damage or result in failure of the antioxidant defence system, leading to increased oxidative stress and free radical damage [1]. As per the World Health Organization (WHO), the global prevalence of WD is 30-100/million [2]. A study conducted in North India reported that WD affected 7.6% of cases of hepatobiliary disorders [3]. A WD clinic in South India reported 15-20 new WD cases with neurological presentation each year [4].

More than 750 mutations in the ATP7 B gene have been reported causing WD to date [5]. A study from South India reported 13 novel mutations among 36 different ATB7 B mutations [5]. In the Chinese population, the p.R778L missense mutation at exon 8 is the most commonly reported, while the p.C271* mutation is most commonly reported in Indians and is reported to cause severe clinical manifestations in the first or second decade of life [6].

The article "Wilson Disease Masquerading as Nephrotic Syndrome: A Case Report" was published in 2025. Journal: Cureus.

The clinical features of WD are heterogeneous, ranging from mild asymptomatic to acute or chronic liver involvement and neuropsychiatric manifestations. A study on 282 Indian patients reported that 70% of cases had initial neurologic manifestations, 15% of cases had hepatic manifestations, and 4% of cases had both hepatic and neurologic manifestations [7]. While neurological and hepatic manifestations are well known, renal manifestations are less commonly seen. The reported renal complications include copper-induced tubular dysfunction, ranging from mild dysfunction to complete Fanconi syndrome, renal calculi, renal tubular acidosis, and acute kidney injury in severe WD [8]. Glomerular injuries as minimal change nephrotic syndrome, membranous nephropathy, and rarely glomerulonephritis, are also reported and can occur due to direct injury due to copper deposition, or as a complication of D-Penicillamine (DPA) therapy [9].

## Case presentation

An eight-year-old boy presented to the pediatric outpatient department with a 15-day history of progressive abdominal distension and decreased urine output. There was an associated decrease in appetite and weight gain, but no nausea, vomiting, cough, or shortness of breath was reported. After around one week, it was followed by progressive swelling of the legs. Clinical examination revealed bilateral pedal edema, ascites, and scleral icterus. His blood pressure was 108/68 mmHg (below the 95th percentile and within normal limits). Anthropometric measurements revealed a weight of 26.8 kg and a height of 135.5 cm. Abdominal examination revealed shifting dullness and a palpable spleen tip. Neurological examination was normal. Urinalysis demonstrated 4+ proteinuria, no RBCs or casts, with a normal lipid profile, suggestive of nephrotic syndrome without dyslipidemia. However, a 24-hour urinary protein was not done due to financial constraints. There was no family history of kidney disease or liver disease. Liver function tests demonstrated elevated bilirubin, transaminitis, and raised gamma-glutamyl transferase (GGT) with a deranged coagulation profile (Table 1).

**Table 1:** Laboratory parameters observed in the patient and their normal ranges.

Laboratory parameter	Observed values	Normal range
Aspartate aminotransferase (U/L)	233	17-59
Alanine aminotransferase (U/L)	154	<50
Alkaline phosphatase (U/L)	395	38-126
Gamma-glutamyl transferase (U/L)	262	15-73
Total bilirubin (mg/dL)	2.9	0.2-1.3
Direct bilirubin (mg/dL)	1.3	0-0.3
Indirect bilirubin (mg/dL)	1.6	0-1.1
Activated partial thromboplastin time (sec)	53.8	25-35
Prothrombin time (seconds)	29.4	11-13.5
International normalized ratio	2.7	0.9-1.4
Serum ceruloplasmin (mg/dL)	9.88	20-40
Serum copper (mcg/dL)	33	70-155
24-hour urinary copper excretion (mcg/day)	536	20-50
Blood urea (mg/dL)	17	14-37
Serum creatinine (mg/dL)	0.3	0.52-1.04
Serum sodium (mg/dL)	134	135-145
Serum potassium (mEq/L)	4	3.5-5.5
Serum chloride (mEq/L)	112	98-107
Total protein (gm/dL)	6.9	6.3-8.2
Serum albumin (gm/dL)	2.4	3.5-5
Serum globulin (gm/dL)	4.4	2.8-3.2
Albumin-globulin ratio	0.5	1.3-1.5
Anti-streptolysin O titer	Negative	-
Anti-hepatitis C virus	Non-reactive	-
Hepatitis B surface antigen	Non-reactive	-
Human immunodeficiency virus	Non-reactive	-
Antinuclear antibody	Negative	-

However, there were no neurological manifestations in the child. Abdominal ultrasound revealed features consistent with chronic liver disease, including splenomegaly (15 cm), gallbladder sludge, moderate ascites, and signs indicative of portal hypertension (Figure 1).

The article "Wilson Disease Masquerading as Nephrotic Syndrome: A Case Report" was published in 2025. Journal: Cureus.

**Figure 1:** Ultrasonography showing liver enlargement, portal vein, and gallbladder sludge. GB, gallbladder; CBD, common bile duct

Slit-lamp examination showed Kayser-Fleischer (KF) rings (Figure 2).

**Figure 2:** Slit-lamp examination showing a Kayser-Fleischer ring (white arrow).

Viral hepatitis markers, antineutrophilic antibody (ANA), and hemolysis workup were negative. Serum ceruloplasmin was markedly reduced, confirming the diagnosis of WD with associated nephrotic syndrome. Serum copper levels were also low, and 24-hour urinary copper excretion was elevated. 

The child was initiated on oral penicillamine (250 mg TID), zinc (50 mg BID), diuretics for edema, hepatic support, and a copper-restricted diet. His urine proteinuria was monitored daily with urine dipsticks, and renal function was repeated to monitor for simultaneous penicillamine-induced renal dysfunction. Although a renal biopsy was not performed due to underlying coagulopathy. On follow-up after two weeks, there was symptomatic improvement with resolution of ascites and proteinuria. Hence, the proteinuria was suspected to be due to copper overload, and corticosteroid was not started for the child. Repeat ultrasound showed hepatomegaly with coarse echotexture, irregular margins, prominent portal vein, and reduced portal flow velocity (20 cm/second), consistent with portal hypertension. He was subsequently started on spironolactone (2 mg/kg/day) in two divided dosages per day and propranolol (1 mg/kg/day). After six weeks, ascites had further reduced, and edema had improved. Repeat ultrasound was consistent with findings of portal hypertension and cirrhosis. Family members were counselled regarding screening for WD in siblings.

The article "Wilson Disease Masquerading as Nephrotic Syndrome: A Case Report" was published in 2025. Journal: Cureus.

## Discussion

Although trientine is increasingly favored as a first-line chelating agent for patients with WD, we opted for penicillamine due to its greater affordability. Penicillamine therapy, however, has been associated with renal adverse effects, particularly glomerular injury leading to nephrotic syndrome. Renal involvement in WD can be due to underlying disease pathology or drug-related (DPA). In WD, underlying copper accumulation can cause either glomerular or non-glomerular (tubular) injury [9]. In 1948, Uzman and Denny-Brown first reported aminoaciduria in a case of WD [10]. In 1959, Litin et al. reported hypercalciuria in a patient with WD [11]. Renal involvement in WD most commonly affects the renal tubules but is not limited to them. These present as renal tubular acidosis, acute tubular necrosis, glycosuria, proteinuria, hypercalciuria, aminoaciduria, hyperphosphaturia, impaired acidification, and hematuria [9]. The tubular dysfunction eventually leads to nephrolithiasis, nephrocalcinosis, and ultimately kidney failure. Our case did not exhibit any of these symptoms. Moreover, neurological and neuropsychiatric manifestations are much common in children with WD presenting with KF ring. In our case, despite the presence of the KF ring, there were no neurological manifestations. Minimal change disease and other common etiologies were considered and ruled out based on the absence of dyslipidemia, normal renal function, and a rapid response to copper chelation without corticosteroids. This supports a direct pathophysiological role of copper.

A cross-sectional study among Chinese individuals with WD demonstrated an increased occurrence of chronic kidney disease (CKD), with a dose-dependent rise in serum copper levels [12]. Glomerular pathology resulting in nephrotic syndrome is more frequently reported as a complication of DPA therapy rather than as an initial manifestation of WD [9]. Case reports also exist of WD presenting as minimal change nephrotic syndrome with accompanying hyperlipidemia [13,14]. Rare case reports exist of WD presenting as nephrotic syndrome, IgA nephropathy, and membranoproliferative glomerulonephritis, with nephrotic-range proteinuria and elevated creatinine, likely due to abnormal deposition of immune complexes in the glomeruli [13-16]. On the other hand, glomerular injury with DPA is frequently reported, and the most common is membranous nephropathy [8,17]. The median time of onset of renal symptoms after starting DPA therapy is reported to be seven months (up to five years), although the earliest reported case is two weeks [8,18]. DPA-induced nephrotic syndrome typically resolves within months after discontinuation but can persist for up to two years [8]. In our patient, DPA therapy was initiated with monitoring of proteinuria and renal function. The treatment led to the resolution of symptoms, and no proteinuria was observed at the two-month follow-up. Long-term follow-up will be needed if the child develops other renal complications of DPA therapy. Nephrotic syndrome is most commonly associated with penicillamine; however, in our case, proteinuria preceded any chelation treatment, and initiation of chelation therapy led to improvement in glomerular function, supporting a potentially reversible copper-mediated glomerulopathy even in the presence of significant proteinuria.

The article "Wilson Disease Masquerading as Nephrotic Syndrome: A Case Report" was published in 2025. Journal: Cureus.

## Conclusions

This report highlights the importance of recognizing nephrotic syndrome as a, though rare, presenting feature of WD in children. Common causes, such as minimal change disease, should be excluded before attributing renal involvement to WD. Renal involvement in WD can present as nephritic or nephrotic syndrome, either as a direct consequence of copper accumulation or as an adverse effect of chelation with DPA. Early recognition of such atypical presentations is critical for early diagnosis and management, particularly in regions with a higher prevalence of WD. This case also contributes to the growing evidence highlighting the diverse clinical spectrum of WD.
